# The Effect and Mechanism of New Processing Method of Codonopsis pilosula on Endocrine Physique Index in Rats

**DOI:** 10.1155/2022/7703612

**Published:** 2022-04-18

**Authors:** Xiaomeng Gong, Changjiang Hu

**Affiliations:** The Ministry of Education Key Laboratory of Standardization of Chinese Herbal Medicine, Key Laboratory of Systematic Research, Development and Utilization of Chinese Medicine Resources in Sichuan Province—Key Laboratory Breeding Base Co-Founded by Sichuan Province and MOST, Sichuan Chengdu 611137, China

## Abstract

**Objective:**

To explore the effect and mechanism of a new processing method of Codonopsis pilosula (CP) on the endocrine physique index in rats.

**Methods:**

The rats were randomly assigned into the control group, model group, CP group (3.75 g/kg crude drug), rice-fried CP group (3.75 g/kg crude drug), and honey-roasted CP group (3.75 g/kg), with 10 rats in each group. All rats were gavaged according to the body weight of 1 mL/100 g every morning for 3 weeks. The water extracts of different processed products of CP were given to the drug group, the blank group, and the model group which were given the same volume of normal saline during the experiment. The model group and each administration group were fed every other day and drank freely for 21 days, during which the weight was weighed every 2 days. The changes of the organ index; the contents of cyclic adenosine monophosphate (cAMP), cyclic guanosine monophosphate (cGMP), adrenocorticotropic hormone (ACTH), and cortisol (Cor); and the activity of sodium and potassium adenosine triphosphate (Na^+^K^+^-ATP) were measured by enzyme-linked immunosorbent assay (ELISA). The expression of aquaporin-1 (AQP1) and aquaporin-2 (AQP2) mRNA was detected by RT-PCR.

**Results:**

Effect on the organ index: the organ index of the control group, CP group, rice-fried group, and honey moxibustion group was higher compared to that of the model group, and the organ index of the honey moxibustion group was the highest (*P* < 0.05). The level of cAMP and the ratio of cAMP/cGMP in the model group were significantly higher compared to those of the control group (*P* < 0.05); CGMP in the model group decreased significantly (*P* < 0.05). Compared with the model group, the level of cAMP in the CP group, rice-fried group, and honey moxibustion group decreased significantly, while the ratio of cGMP and cAMP/cGMP increased significantly (*P* < 0.05). Compared with the CP group, rice-fried group, and honey moxibustion group, the level of cAMP and the ratio of cAMP/cGMP in the honey moxibustion group were lower compared to those in the other two groups, and the ratio of cGMP in the honey moxibustion group was higher compared to that in the other two groups (*P* < 0.05). The contents of ACTH and Cor in the model group were significantly higher compared to those in the control group (*P* < 0.05). Compared with the model group, the contents of ACTH and Cor in the CP group, rice-fried group, and honey moxibustion group were significantly lower compared to those in the model group (*P* < 0.05). Compared with the CP group, rice-fried group, and honey moxibustion group, the contents of ACTH and Cor in the honey moxibustion group were higher compared to those in the other two groups (*P* < 0.05). The content of the Na^+^K^+^-ATP enzyme in the model group was significantly higher compared to that in the control group (*P* < 0.05). Compared with the model group, the content of the Na^+^K^+^-ATP enzyme in the CP group, rice-fried group, and honey moxibustion group decreased significantly (*P* < 0.05). Compared with the CP group, rice-fried group, and honey moxibustion group, the content of the Na^+^K^+^-ATP enzyme in the honey moxibustion group was higher compared to that in the other two groups (*P* < 0.05). The expression of AQP1 and AQP2 mRNA in the kidney tissue of the kidney yin deficiency model group was significantly higher compared to that of the control group (*P* < 0 05). Compared with the model group, the expression levels of AQP1 and AQP2 mRNA in the renal tissue of rats in the CP group, rice-fried group, and honey moxibustion group decreased in different degrees (*P* < 0.05). There was no statistical difference between the CP group, rice stir-frying group, and honey moxibustion group.

**Conclusion:**

This study proves that the new processing method of CP can improve the endocrine physique index of rats, enhance their organ quality, and regulate the disorder of water metabolism in kidney yin deficiency syndrome and has a certain therapeutic effect on kidney yin deficiency syndrome. Different new processing methods of CP have different effects on promoting endocrine physique indexes of rats. It is concluded that honey-roasted CP has the best effect on promoting spleen deficiency, which may be through glucose metabolism, amino acid metabolism, and nucleotide metabolism, increasing ATP energy metabolism, so as to strengthen the symptoms of spleen deficiency in rats. The experimental data of this study indicate that the effect of honey-roasted CP is better compared to that of other processed products, which provides an experimental basis for the rational clinical application of the new processed products.

## 1. Introduction

Codonopsis pilosula (CP) is a classical tonic traditional Chinese medicine (TCM), which is widely distributed [1]. According to the Chinese Pharmacopoeia, Codonopsis pilosula (Franch.) Nannf. is the dried root of CP, CP, and CP in Campanulaceae [2]. It is recorded in ancient documents such as the *Materia Medica from Xin*, *Compendium of Materia Medica*, and *Textual Research on Plant Names*. CP is sweet and flat, which belongs to the spleen and lung meridian, which can strengthen the spleen and lung, tonify the middle, and benefit qi. Clinically, it is mainly adopted for general weakness, less food, dry mouth, long diarrhea, prolapse of the anus, and other symptoms, such as weakness of the spleen and stomach and deficiency of qi and the blood, with the effects of moistening the lung and resolving phlegm and nourishing yin and the stomach. CP was first produced in ancient Luzhou (present-day Jincheng and Changzhi City) and is one of the famous “four northern medicines” with a long history of use and good quality [3]. It is a commonly adopted TCM for tonifying both qi and the blood, and the content of ancient processing is relatively simple. It was recorded in the Qing Dynasty, and the processing methods of fried rice and honey-fried CP were perfected in modern times. The processing methods of fried CP have been also developed, such as stir-frying with bran and soil. The 2015 edition of Pharmacopoeia included fried CP and stipulated its processing methods [4]. CP is good at invigorating fluid and benefiting qi, which is mainly adopted for deficiency of both qi and the blood, injury of both fluid and qi, and other syndromes. Fried CP with rice can enhance the effect of tonifying qi and invigorating the spleen, which is mostly adopted for weakness of the spleen and stomach, less food, and sparse stool. Honey-broiled CP focuses on tonifying qi, moistening dryness, and nourishing yin with an obvious effect on shortness of breath, visceral prolapse, and irregular menstruation [4, 5]. Based on the drug efficacy, the functional indications are different after processing, indicating that the content of its components has changed, but so far, its content has not been stipulated in the Pharmacopoeia and local standards. There are a variety of processing methods of CP, and different processing methods have great influence on the chemical composition of CP [5]. The effect of CP on invigorating the spleen is enhanced after fried rice, and the effect of invigorating qi of CP is enhanced after honey roasting. Wine and honey broiling can increase the content of polysaccharides of CP, while fried rice and bran can reduce the content of pol [5, 6]. Some scholars have pointed out that different processed products of CP have shown that honey-fried CP is better than fried CP and raw CP in improving the phagocytosis of macrophages in mice [6]. However, the mechanism of its qi-invigorating effect has not been reported. At present, there are related reports on the effect of CP on promoting the exercise-induced fatigue ability of mice, but the effect and mechanism of different processed products on spleen deficiency caused by fatigue have not been reported [6, 7].

Processing is one of the means to enhance the curative effect of TCM [6]. The clinical use of raw CP is often for spleen and lung weakness, shortness of breath, palpitation, deficient asthma cough, and other diseases. When fried in rice, CP smells fragrant and enhances the effect of invigorating qi and invigorating the spleen [7]. Honey-roasted CP has a slow sexual taste, and the effect of tonifying the middle and replenishing qi is stronger compared to raw codon. Soil frying can enhance the effect of CP on invigorating the spleen and stopping diarrhea, while bran frying emphasizes the role of CP in the stomach. Some scholars used the carbon particle clearance test and antifatigue experiment to compare the qi-replenishing effect of CP, fried CP with rice, and CP with honey [7, 8]. The experiment preliminarily proved that the clinical effect of CP with honey was the best. This experimental study further proved that the effect of honey-broiling CP on invigorating the spleen and replenishing qi was better compared to that of CP. Some scholars have found that fried CP can enhance the contraction and relaxation of the gastrointestinal smooth muscle [8]. It is speculated that it is one of the mechanisms of rice frying to promote the efficacy of CP in invigorating the spleen and replenishing qi. Studies have indicated that fried dried CP with rice soup can significantly enhance the degree of hypoxia tolerance and swimming time in mice, so its antistress effect is significantly better compared to that of raw CP [8, 9]. Wang et al., when studying the effect of processing on the curative effect of TCM compound prescription, found that when Shenling Baizhu powder was used to improve the immunity of the body, the raw products of CP, licorice, Atractylodes macrocephala, and Atractylodes macrocephala and Coix seed had the best effect; in promoting the digestion and absorption of patients with spleen deficiency and diarrhea, Shenling Baizhu Powder, which was composed of fried bran products of CP and licorice, yam, and Coix seed, had the best effect [9]. Liujunzi decoction is a good prescription for invigorating the spleen and replenishing qi. In recent years, it is mainly adopted in the treatment of digestive tract diseases. Some studies have indicated that the effect of CP, tangerine peel, Atractylodes macrocephala, and Pinellia ternata in the treatment of digestive tract reaction is significantly better compared to that of raw products [10]. CP is a commonly adopted bulk medicinal material, its processing methods are varied, and different processing methods have great changes in its effective components and efficacy. In view of this, this study focuses on the improvement effect and mechanism of the new processing method of CP on the endocrine physique index of rats, and the results are reported as follows.

## 2. Materials and Methods

### 2.1. Materials

CP slices (batch number: 20180104), fried CP slices (batch number: 20180110), and honey-fried CP slices (batch number: 20180101) are provided by the Shanxi Zhendong Group, all of which are CP and its processed products.

### 2.2. Instrument

The instruments we used in this study were as follows: Centrifuge; Multiskan FC enzyme labeling instrument (American Thermo company); gel imager (British Uvitec Ltd., model: Alliance Q9); electrophoresis instrument, electrophorester, and electrophoresis slot (Bole Bio-Rad, model: BE6085); shaker (Kylin-Bell Lab Instruments Co., Ltd., model: 7s-8s); and analytical balance (Shanghai Yueping Scientific instrument Manufacturing Co., Ltd.).

### 2.3. Animal

The animals used in the study are 50 SPF SD rats, half male and half female, obtained from the Shanghai Shrek Experimental Animal Co., Ltd. (animal production license number: SCXK (Shanghai) 2007-0005).

### 2.4. Methods

#### 2.4.1. Animal Grouping, Modeling, and Administration of SD

The rats were fed adaptively for 7 days (temperature 25°C, humidity 50 ± 10%, alternating light and dark for 12 hours). 50 SD rats were enrolled and assigned into the control group, model group, CP group (3.7 5g/kg crude drug), rice-fried CP group (3.75 g/kg crude drug), and honey-roasted CP group (3.75 g/kg) with 10 rats in each group. All rats were gavaged according to 1 mL/100 g body weight every morning for 3 weeks. The water extracted from different processed products of CP were given intragastrically in the administration group, and the same volume of normal saline was given to the blank group and the model group. One hour after administration every day, all rats (except the control group) were loaded with 10% lead and placed in a circular tank with a water temperature of 25 ± 1°C to swim until the rats sank to the bottom and did not surface within 10 seconds, and the exhaustive swimming ended. During the experiment, the model group and each administration group were fed every other day and drank freely for 21 days, during which the weight was weighed every 2 days. After intragastric administration for 1 hour on the last day, the rats were weighed and exhaustive swimming was carried out, and the exhaustion time of rats in each group was recorded. The rats were removed from the swimming tank, dried with a dry towel, and injected intraperitoneally with 20% uratan (0.75 mL/100 g body weight). The rats were anesthetized, and the blood was taken from the abdominal aorta quickly. The rats underwent 13000 rpm 15 min centrifugation for 1 hour; the supernatant was taken and stored at -20°C. The right leg muscle (gastrocnemius muscle) tissue of all rats was stripped and stored at -80°C.

#### 2.4.2. Determination of Serum Biochemical Indexes

The serum biochemical indexes were measured by cAMP kit (E20190317-30440A), cGMP kit (E2019031-30439A), ACTH kit (E20190314-30276A), Cor kit (E20190308-30678A), sodium-potassium-adenosine triphosphate (Na+K+-ATP) enzyme-linked immunosorbent assay (ELISA) kit (E-2019031-34351A). In addition, whole protein extraction kit, BCA protein concentration determination kit, ECL chemiluminescence detection kit, rainbow 245 broad-spectrum protein MarKer, and SDS-PAGE gel preparation kit were applied (Beijing Solebao Technology Co., Ltd., product numbers: BC3711, PC0020, SW2010, PR1920, and P1200-2, respectively).

#### 2.4.3. Muscle Sample Preparation

200 mg of muscle tissue was excised (on ice), homogenised at 4°C for 15  min, and centrifuged at 13,000 r/min. The supernatant was transferred to a 5 ml EP tube, blown dry with nitrogen, and centrifuged at 13,000 r/min for 20 min at 4°C. The supernatant was stored at -20°C for measurement. The liver, spleen, lungs, and bilateral kidneys of the rats were also isolated, washed with saline, dried with filter paper, and weighed.

### 2.5. Index Measurement

In strict accordance to the method provided by the kit instructions, the contents of cAMP, cGMP, ACTH, and Cor in the rat serum and the activity of the Na^+^K^+^-ATP enzyme in the rat plasma were determined, and the expression of AQP1 and AQP2 mRNA was detected by the RT-PCR method. Organ index measurement: the organ mass was measured by analytical balance and calculated according to “organ index = (organ mass/body mass) × 1000.”

### 2.6. Statistical Analysis

Using SPSS 21.0 statistical software, before statistical analysis, the measurement data were tested by normal distribution and variance homogeneity analysis to meet the requirements of normal distribution or approximate normal distribution. The data was expressed as $\bar{x}\pm s$. The repeated measurement data were analyzed by repeated measurement analysis of variance. Additionally, multiple groups were compared by one-way ANOVA analysis *t*-test was employed to compare the two groups, *n* (%) was employed as an example to represent the counting data, and the *χ*^2^ test was employed to indicate that the difference was statistically significant (*P* < 0.05).

## 3. Results

### 3.1. Effects of Different Processed Products on Organ Index in Rats with Kidney Yin Deficiency

Effect on organ index: the organ index of the control group, CP group, rice-fried group, and honey moxibustion group was higher compared to that of the model group; comparing the CP group, rice-fried group, and honey moxibustion group, the organ index of the honey moxibustion group was the highest (*P* < 0.05). All the data results are indicated in Table 1.

### 3.2. Effect on cAMP, cGMP, and cAMP/cGMP

The level of cAMP and the ratio of cAMP/cGMP in the model group were significantly higher compared to those in the control group (*P* < 0.05); cGMP in the model group decreased significantly (*P* < 0.05). Compared with the model group, the level of cAMP in the CP group, rice-fried group, and honey moxibustion group decreased significantly, while the ratio of cGMP and cAMP/cGMP increased significantly (*P* < 0.05). Comparing the CP group, rice-fried group, and honey moxibustion group, the level of cAMP and the ratio of cAMP/cGMP in the honey moxibustion group were lower compared to those in the other two groups, and the ratio of cGMP in the honey moxibustion group was higher compared to that in the other two groups (*P* < 0.05). All the data results are indicated in Table 2.

### 3.3. Effect on the Content of ACTH and Cor

The contents of ACTH and Cor in the model group were significantly higher compared to those in the control group (*P* < 0.05). Compared with the model group, the contents of ACTH and Cor in the CP group, rice-fried group, and honey moxibustion group were significantly lower (*P* < 0.05). Comparing the CP group, rice-fried group, and honey moxibustion group, the contents of ACTH and Cor in the honey moxibustion group were higher compared to those in the other two groups (*P* < 0.05). All the data results are indicated in Table 3.

### 3.4. Effect on Na^+^K^+^-ATP Enzyme Content

The content of the Na^+^K^+^-ATP enzyme in the model group was significantly higher compared to that in the control group (*P* < 0.05). Compared with the model group, the content of the Na^+^K^+^-ATP enzyme in the CP group, rice-fried group, and honey moxibustion group decreased significantly (*P* < 0.05). Comparing the CP group, rice-fried group, and honey moxibustion group, the content of the Na^+^K^+^-ATP enzyme in the honey moxibustion group was higher compared to that in the other two groups (*P* < 0.05). All the data results are indicated in Table 4.

### 3.5. Effects of AQP1 and AQP2 mRNA Expression in Renal Tissue of Rats in Different Groups

The expression of AQP1 and AQP2 mRNA in the kidney tissue of the kidney yin deficiency model group was significantly higher compared to that of the control group (*P* < 0.05). Compared with the model group, the mRNA expression levels of AQP1 and AQP2 in the renal tissue of rats in the CP group, rice-fried group, and honey moxibustion group were significantly lower compared to those in the model group (*P* < 0.05); no statistical difference was exhibited between the blank group and the blank group. All the data results are indicated in Figure 1.

## 4. Discussion

The authentic CP are included in the 2015 edition of the Chinese Pharmacopoeia: Modesta (Nannf.) L.T.Shen and Sichuan CP Codonopsis tangshen Oliv [10]. At present, CP is mainly planted to be sold in the market, and the production areas are distributed in Yunnan, Henan, Northeast, Ningxia, North China, and Shaanxi, among which Shaanxi has the highest quality. CP is mainly produced in northwest Sichuan and Gansu, Qinghai, Shaanxi, and other places. CP is produced in western Hubei, northwest Hunan, northeast Sichuan, and northern Guizhou. In addition, there are C. clematidea (CP), C. subglobosa (CP), C. nervosa (CP), C. macrocalyx (CP), C. thalictrifolia var. mollis (CP), C. viridiflora (green CP), and Codonopsis lanceolata (C. pilosula var. volubilis), most of which are wild products, which have not been well developed and utilized at present. CP, which is similar to most of TCM, has complex ingredients [11, 12]. In recent years, the chemical constituents of CP have been deeply studied. It is found that there are mainly sugars, phenylpropanoids, and terpenes. Carbohydrate is one of the effective components of CP, which has the effects of enhancing immunity, antioxidation, and antitumor. It is mainly assigned into polysaccharides and monosaccharides, which include inulin, fructose, *α*-D-fructose hexanol, and *β*-D-glucose hexanol. CP is rich in triterpenes and sesquiterpenes, including Atractylodes lactone II, Atractylodes lipid III, dandelion terpenol, dandelion terpenol acetate, cork ketone, and other compounds [13]. Phenylpropanoid compounds are isolated from CP, which are also the main active components, such as syringin, Codonopsis ginsenoside I, Codonopsis ginsenoside II, Codonopsis ginsenoside III, and Codonopsis ginsenoside IV. Codonopsis alkyne (lobetyolin) is one of the characteristic components of CP, which has a variety of physiological activities, such as anti-inflammatory, anticancer, and immunomodulatory activities [14]. Codonopsis alkynes are also one of the active components of CP protecting gastric mucosa [15]. In addition, CP also includes various sterols and alkaloids. CP is a commonly used traditional tonifying medicine in TCM. Modern studies have indicated that CP contains a variety of chemical components, which can enhance immunity, dilate blood vessels, reduce blood pressure, promote microcirculation, and enhance hematopoiesis [16].

By detecting the phagocytic activity of mouse macrophages, Jiao et al. proved that CP can significantly promote the phagocytic activity of mouse macrophages and CP can strengthen the immunity of the body from the cellular level [17]. Wang et al. also confirmed that CP can increase the content of interleukin-2 (IL-2) in serum of aging mice from the level of cytokines, so it can enhance the immunity of mice and enhance their antiaging ability [18]. The antioxidant function of CP is mainly reflected in regulating the activity of antioxidant enzymes. Shori et al. believe that CP can resist oxygen free radicals, is a strong antioxidant, and plays an important role in delaying aging [19]. Li et al. also proved that Xinjiang CP polysaccharides can delay human aging by increasing the activity of superoxide dismutase (SOD) in the human body. Subcutaneous injection of the water extract of CP could significantly increase the number of red blood cells and the content of hemoglobin in rabbits and increase the blood concentration [20]. When combined with compound medicine, CP can inhibit the synthesis of thromboxane B2 in plasma and counteract the phenomenon of platelet aggregation caused by coronary heart disease or angina pectoris. In addition, CP can reduce erythrocyte sclerotic index, increase blood fluidity, promote human microcirculation, and significantly inhibit the formation of thrombus in vitro [21]. In addition, CP may also reduce blood pressure by dilating blood vessels and increasing the output of the heart, brain, viscera, and other organs [22]. The pharmacological activity of TCM polysaccharides is obvious, among which CP polysaccharides can protect gastric tissue, increase pepsin activity and excretion, increase intestinal peristalsis, and promote digestion. Its mechanism can increase the activity of SOD in serum and tissue, decrease the content of malondialdehyde (MDA) in serum and tissue, regulate the activity of glutathione peroxidase (GSH-Px) in gastric tissue, and protect gastric tissue [23]. In addition to the above effects, CP can also prolong the sleep time caused by ether and pentobarbital sodium, strengthen the antistress ability of mice, but also have anti-inflammatory and analgesic effects [24].

The processing of medicinal materials is an important part of TCM culture. The processing of CP began to be recorded in the Qing Dynasty [25]. In modern times, it inherited fried CP (“current disease”) and honey-fried CP (“Zhiquan”) and developed processing methods such as stir-frying, rice soup, and steaming [25, 26]. The 2015 edition of the Pharmacopoeia included the processing method of fried CP and stipulated its method. CP is rich in volatile oil. In the process of heating and processing, the volatile oil with low boiling point volatilizes a lot and loses a lot. Therefore, the volatile oil content of fried CP with rice and bran is lower compared to that of raw CP [26]. Stir-frying is the simplest processing method of CP, and the time and heat of frying have a significant effect on the quality of CP. The research shows that with the deepening of stir-frying, the degree of internal dissociation of CP becomes larger and H^+^ increases, which leads to the decrease of pH of CP, so the pH of raw CP, fried CP, and CP decreases in turn. Meanwhile, HPLC found that with the deepening of frying, the peak of CP disappeared [27]. Sulfur fumigation is one of the common processing methods of TCM. After sulfur fumigation, it is found that the content of alkynyl glycosides in CP decreased significantly, while the content of total flavonoids increased significantly. Recent research found that after CP was fried with soil, the contents of Fe, Li, Ca, Zn, Mn, and Sr were much higher than those of raw products and other processed products [28]. It is also found that the content of the Cu element in Radix Codonopsis is higher compared to that in other processed products, while the content of the Li element was lower compared to that of other processed products. 5-HMF is an aldehyde compound obtained by dehydration of glucose at high temperature. The results indicated that the content of 5-HMF in CP was not significantly changed by bran stir-frying, soil-broiling, and wine-broiling, but the content of 5-HMF in CP was significantly increased by honey. Other scholars further explored the processing mechanism of CP by the HPLC method and compared the chemical composition changes of CP before and after fried rice [29]. It is found that 5-HMF was newly formed in CP after fried rice, and the content of Codonopsis polysaccharides decreased gradually with the increase of the 5-HMF content, which suggested that processing might promote the transformation of Codonopsis polysaccharides to 5-HMF. The content of extract is also one of the indexes of the quality standard of TCM. The results indicated that the contents of extracts in CP and its processed products were in the following order: honey broth > wine broth > metric system > raw product > soil stir-fry. The content of effective components of CP changed after processing, which provided a material basis for the changes of pharmacodynamics of different processed products.

CP is a commonly employed health medicine with high medicinal value, high dosage, and wide clinical application. In recent years, CP has made great progress in promoting immunity and delaying aging. In addition, with the improvement of living standards, people attach importance to the health care function of CP [28, 29]. The study on the active components and pharmacodynamic effects of CP is beneficial to clarify its efficacy mechanism and lay a scientific foundation for the development of CP medicinal materials and medicinal resources. Cyclic nucleotides are the main substances that regulate cell function and activity. Under normal conditions, the levels of cAMP and cGMP in serum do not change, but when the body continues to be excited, the level of cAMP increases and the ratio of cAMP/cGMP increases, indicating that the metabolism of the body is affected and the basic metabolism is enhanced. The rats with kidney yin deficiency indicated hyperfunction of the hypothalamus-pituitary-adrenal (HPA) axis, which was mainly characterized by the increase of the level of corticotropin, which stimulated the release of cortisol from the adrenal cortex, so ACTH and Cor were employed as indicators to detect the state of rats [30]. Thyroid is the largest secretory gland in the human body; thyroxine can promote substance and energy metabolism. When thyroxine in the body is beyond the normal range, the activity of the Na^+^K^+^-ATP enzyme in the heart, liver, and other tissues increases significantly. According to this, rats are given levothyroxine sodium and reserpine suspension to make rats indicate the symptoms of kidney yin deficiency in TCM [31]. CP has the effect of nourishing yin and tonifying the kidney, and rats with kidney yin deficiency are treated. By observing the clinical indexes of rats with kidney yin deficiency, it was found that they lost weight and are easily frightened and irritable, and there were significant changes after treatment in each group of CP, indicating that Ligustrum lucidum has a therapeutic effect on the symptoms of kidney yin deficiency. The traditional theory of TCM says that “the kidney dominates water,” and the kidney belongs to water in the five elements, which plays an important role in regulating the metabolic balance of human body fluid [31, 32].

In recent years, aquaporins are mostly employed to study the regulatory mechanism of water absorption, secretion, and excretion, in which AQP1 and AQP2 are closely related to kidney regulation of water reabsorption and play an important role in water-liquid balance and osmotic pressure regulation. The results of Western blot indicated that the expression of AQP1 and AQP2 in the kidney tissue of the kidney yin deficiency model group increased, and the expression of AQP1 and AQP2 decreased after treatment with various processed products of CP, indicating that CP can regulate the levels of AQP1 and AQP2 in the kidney and plays a positive role in the disorder of water metabolism in kidney yin deficiency syndrome [32]. This study proves that different processed products of CP can promote the hormone level of hyperthyroidism rats with kidney yin deficiency, strengthen their organ quality, regulate the disorder of water metabolism in kidney yin deficiency syndrome, and have a certain therapeutic effect on kidney yin deficiency syndrome. CP has the medicinal characteristics of nourishing the liver and kidney. After processing, the effect of regulating the hormone level of kidney yin deficiency syndrome is better, the organ quality of the body is enhanced obviously, and the disorder of water and fluid metabolism is promoted.

Conclusively, this study proves that the new processing method of CP can enhance the endocrine physique index of rats, promote their organ quality, regulate the disorder of water metabolism in kidney yin deficiency syndrome, and have a certain therapeutic effect on kidney yin deficiency syndrome. CP has the medicinal characteristics of nourishing the liver and kidney. After processing, the effect of regulating the hormone level of kidney yin deficiency syndrome is better, the organ quality of the body is strengthened obviously, and the disorder of water and fluid metabolism is enhanced. Different new processing methods of CP have different effects on promoting endocrine physique indexes of rats. It is concluded that honey-roasted CP has the best effect on improving spleen deficiency, which may be through glucose metabolism, amino acid metabolism, nucleotide metabolism, and increased ATP energy metabolism, so as to enhance the symptoms of spleen deficiency in rats. The experimental data of this study indicate that the effect of honey-roasted CP is better compared to that of other processed products, which provides an experimental basis for the rational clinical application of the new processed products.

## Figures and Tables

**Figure 1:** Expression of AQP1 and AQP2 mRNA in different groups.

**Table 1:** Effects of different processed products on organ index of rats with kidney yin deficiency ($\bar{x}\pm s$, mg·g^−1^).

Group	Kidney	Liver	Spleen
Control group	13.58 ± 1.66^∗^	56.69 ± 2.43^&^	4.52 ± 0.31^￥^
Model group	9.49 ± 2.21^∗^	35.66 ± 2.21^&^	1.46 ± 0.31^￥^
CP	11.48 ± 1.21^∗^	44.67 ± 3.41^&^	2.46 ± 0.16^￥^
Rice-fried formation	11.55 ± 1.21^∗^	44.77 ± 3.12^&^	2.47 ± 0.18^￥^
Honey moxibustion group	12.78 ± 1.24^∗^	45.77 ± 1.25^&^	3.41 ± 1.21^￥^
*P*	<0.05	<0.05	<0.05

Indication: ^∗^*P* < 0.05, ^&^*P* < 0.05, ^￥^*P* < 0.05.

**Table 2:** Effects of different processed products on cAMP, cGMP, and their ratio in rats with kidney yin deficiency ($\bar{x}\pm s$).

Group	cAMP (nmol·L^−1^)	cGMP (nmol·L^−1^)	cAMP/cGMP
Control group	32.66 ± 1.31^∗^	29.44 ± 1.45^&^	1.16 ± 0.11^￥^
Model group	51.66 ± 2.44^∗^	19.45 ± 2.85^&^	2.75 ± 0.33^￥^
CP	44.54 ± 2.22^∗^	22.67 ± 1.56^&^	2.31 ± 0.15^￥^
Rice-fried formation	44.54 ± 2.12^∗^	23.56 ± 1.77^&^	2.21 ± 0.11^￥^
Honey moxibustion group	42.78 ± 1.24^∗^	26.63 ± 1.25^&^	1.78 ± 0.42^￥^
*P*	<0.05	<0.05	<0.05

Indication: ^∗^*P* < 0.05, ^&^*P* < 0.05, ^￥^*P* < 0.05.

**Table 3:** Effects of different processed products on the contents of ACTH and Cor in rats with kidney yin deficiency ($\bar{x}\pm s$, nmol·L^−1^).

Group	ACTH	Cor
Control group	17.42 ± 2.42^∗^	10.45 ± 0.52^&^
Model group	35.66 ± 1.44^∗^	16.64 ± 2.56^&^
CP	20.54 ± 2.12^∗^	12.14 ± 1.77^&^
Rice-fried formation	20.77 ± 2.31^∗^	12.18 ± 1.56^&^
Honey moxibustion group	22.78 ± 1.24^∗^	14.63 ± 1.12^&^
*P*	<0.05	<0.05

Indication: ^∗^*P* < 0.05, ^&^*P* < 0.05.

**Table 4:** Effects of different processed products on the content of Na^+^K^+^-ATP enzyme in rats with kidney yin deficiency ($\bar{x}\pm s$).

Group	Na^+^K^+^-ATP enzyme
Control group	19.42 ± 1.46^∗^
Model group	30.75 ± 2.56^∗^
CP	21.77 ± 2.53^∗^
Rice-fried formation	22.74 ± 2.12^∗^
Honey moxibustion group	24.77 ± 1.32^∗^
*P*	<0.05

Indication: ^∗^*P* < 0.05.

## Data Availability

No data were used to support this study.
